This article has been retracted.

# Efficacy of Glucocorticoids and Glucocorticoid-Induced Hyperglycaemia in Renal Disease: A Meta-Analysis of Randomized Controlled Trials

**DOI:** 10.1155/2022/2484626

**Published:** 2022-03-07

**Authors:** Zeng Wang, Yi Qian Qu, Yang Zhang, Xing Yu Zhu, Xiao Wei Gong, Hong Yu Chen

**Affiliations:** ^1^Hangzhou Traditional Chinese Medicine Hospital Affiliated to Zhejiang Chinese Medical University, Hangzhou, Zhejiang, China; ^2^College of Basic Medical Science, Zhejiang Chinese Medical University, Hangzhou, Zhejiang, China; ^3^Baiyang Community Health Service Center, Baiyang Street, Hangzhou, Zhejiang, China

## Abstract

**Background:**

Glucocorticoids are the most effective anti-inflammatory and immunosuppressive drugs used to treat patients with renal disease. This study pooled the current evidence of the efficacy of Glucocorticoids and Glucocorticoid-induced hyperglycaemia in renal disease.

**Methods:**

We conducted a systematic literature search on PubMed, Cochrane Central, and Web of Science for relevant randomized controlled trials (RCTs) up to September 1, 2021. The meta-analysis, sensitivity analysis and bias analysis were performed using Review Manager 5. 3.

**Results:**

In this study, seven RCTs with 797 patients were included in our analysis. The analysis revealed that glucocorticoids had a certain alleviating effect on the reduction of renal function. (risk ratio [RR] 0.49 95% confidence interval [Cl] 0. 28 to 0.85, p =0.01) and reduction of proteinuria (weight mean difference [WMD] -0.43; 95% CI -0.57 to-0.28) when compared with the control group. Patients receiving glucocorticoids therapy did not have an increased risk of developing new-onset diabetes mellitus or impaired glucose tolerance. (RR 3.76 95% CI 0.54 to 26.10, p =0.18). For other safety outcomes, glucocorticoids therapy did not increase risk of respiratory infections (RR 1.63, 95% CI 0. 69to3. 89, p =0.27) and Gastrointestinal SAEs is relatively controversial (RR 1.10, 95% CI 0.32 to 3.79, p =0.88). *Discussion*. In conclusion, current clinical evidence indicates that glucocorticoids is efficacious and safe to renal disease compared with control. Further research comparing long-term glucocorticoids use is needed.

## 1. Introduction

Glucocorticoids are highly conserved vertebrate hormones that mediate a suite of functional responses to changing conditions over various time scales [1–2]. They are the most effective anti-inflammatory drugs used to treat patients with several disease because of their anti-inflammatory and immunosuppressive properties. Under normal physiological conditions, glucocorticoids control secretion through the hypothalamic-pituitary-adrenal axis, and regulate the normal metabolism of substances in the body [3]. When secretion is insufficient, it shows metabolic disorders. When the human body changes suddenly in the internal and external environment can stress secretion of a large number of glucocorticoids [4]. When the dose is higher than the physiological dose, it can produce immunosuppression and decrease the inflammatory response and other pharmacological effects [5]. It was suggested that glucocorticoids can affect about 20% of human genes to be induced or suppressed during transcription through their exclusive glucocorticoid receptors [6].

In the pathogenesis of several renal disease, hyperactivity or low immunity is the main reason. The pathological manifestations are mainly immune complex deposition, which leads to inflammatory reaction, inflammatory cell infiltration and cell proliferation. Without some supporting therapies including decreasing blood pressure, reducing lipid, glucocorticoids are used to control the progression of renal dysfunction in patients with renal disease [7]. At present, most clinical use is empirical, prone to unreasonable dosage, high incidence of adverse reactions and complications, which affect the clinical treatment effect. And some randomized controlled trials (RCTs) of glucocorticoid therapy for nephropathy show that it can slow the deterioration of renal function and reduce the proteinuria. Meanwhile, the therapy may bring some adverse events. However, the efficacy of glucocorticoids and Glucocorticoid-induced hyperglycaemia in renal disease are still obscure, which is worthy to be confirmed by a large sample of clinical studies.

Using meta-analytical techniques, the present study summarize available evidence from RCTs and estimate the efficacy and safety of glucocorticoid use for the treatment of nephropathy.

## 2. Methods

### 2.1. Search Tragedy

Two authors performed a systematic search of PubMed, Web of Science and Cochrane Library for English-language studies up to September 1, 2021. The following medical subject heading terms and text words were used: Glucocorticoid, Glucorticoid, hydrocortisone, prednisone, prednisolone, triamcinolone, dexamethasone, cortisone, Methylprednisolone, Betamethasone, Beclomethasone, nephropathy, Kidney Diseases, and Diabete, glycuresis, Blood glucose. Another two authors analyzed the titles and abstracts of the articles and ascertained conformity with the inclusion criteria.

### 2.2. Citation selection

All articles after the first screening were further selected by other researchers. Titles and abstracts are independent and carefully selected. The full text is available if the study meets the inclusion criteria.

Inclusion criteria

- the study was a clinical randomized control trial (RCT);
- the study compared glucocorticoid agents (any dose, type) versus placebo/no treatment
- the study have sufficient inspection indicators

Exclusion criteria

- Not randomized
- Studies with any other immunosuppressive agents
- Lack of outcome measures or comparable results

Manually search the bibliography for each selected article to identify other articles that meet the selection criteria.

### 2.3. Data Extraction

Data were extracted by authors from all included trials in accordance with patient characteristics of the study sample, the study drugs, doses, dosage and administration, baseline characteristics of the trials, follow-up and lost at follow-up (%) and the following reported outcomes: (i) the primary outcome was renal survival (defined as renal impairment to the point of doubling serum creatinine or/and achieving ESRD requiring dialysis or transplantation at any time during treatment); (ii) the secondary outcome was New-onset diabetes mellitus or impaired glucose tolerance; (iii) other adverse events of treatment. For consistency, we collected all the analytical data. The clinical characteristics of each study were summarized.

### 2.4. Quality Assessment

To further quantify the literature quality evaluation, Modified Jadad Score [8] has been used to assess reported randomization, blinding, withdrawals, dropouts, inclusion/exclusion criterion, AEs and the statistical analysis. We allocation concealment and intention-to-treat analysis, blinding of investigators, participants and outcome assessors, and completeness to follow up. In addition, to assess publication bias, Egger's test and Begg's funnel plot would be performed if necessary. RevMan5. 3 was used to assess risk from compliance problems and attention bias.

### 2.5. Statistical Analysis

Relative risk (RR) measures were used to analyze dichotomous data from individual trials. For continuous output, the mean and 95% confidence interval (CI) of individual trials are calculated. We calculated RR and CI by Revman5. 3. Statistical heterogeneity was assessed by Cochran's Q statistic and I^2^ statistics. When there is no statistical heterogeneity and when significant heterogeneity is defined as I^2^>50% or Chi squared test p <0.1, the fixed-effect model was used to summarize the study; otherwise, the random effect model was used. For single trials with no events in one or two groups, a continuity correction of 0.5 was added to each cell [9–10].

## 3. Results

### 3.1. Trial Flow and Study Characteristics

The combined search of PubMed, Scientnet, and the Cochrane Library, including some manual searches of related kidney journals, yielded 251 citations. After discarding a number of duplicates retrieved by individual searches, 237 studies were included. After reviewing all titles and abstracts, 223 studies were excluded because they were not RCTs, or were irrelevent, or were animal experiment and so on. Thirteen articles were reviewed in full text to further assess their eligibility; six studies were excluded, because one was unrelated topic, five did not have placebo or suitable control group. Overall, 7 trials had been enrolled in this study [11–17].

Figure 1 and Table 1 summarizes the interventions, population baseline characteristics, study duration, concomitant medications, follow-up, and renal function outcomes in the randomized controlled trials we analyzed.

DRF = Deteriorated renal function; IgAN = Immunoglobulin A nephropathy; UPCR = urine protein to creatinine ratio.

### 3.2. Quality Assessment

A quality assessment of the primary studies is summarized in Table 2. The Jadad scores ranged from 0 to 7 points. The quality of the research was generally mediocre; 3 of 7 studies had a Jadad score of 7, 6 of 7 had a Jaded score of ≥4. Participants and investigators were blinded in only 3 of 7 trials, sufficient details of drop-outs and withdrawals were described in 6 trials.

### 3.3. Effect on Renal survival

Four studies reported the number of renal deterioration. According to our meta-analysis, although the effect of dosage form was not taken into account, it could still be seen that glucocorticoids had a certain alleviating effect on the reduction of renal function. (4 trials, 95% CI 0.28 to 0.85, p =0.01 Figure 2).

No heterogeneity of the effects was found, so univariate study-level meta-regression were not used for heterogeneity analysis.

### 3.4. Effects on Daily proteinuria

5 studies of 7 RCTs assessed daily proteinuria in 578 patients, 284 in the treatment group and 294 in the control group. Overall, according to this analysis, glucocorticoid treatment reduced proteinuria more than the control group (95% CI -0.57 to -0.28, p <0.00001, I^2^ = 79% Figure 3).

### 3.5. Effect on blood glucose

Three studies involved new-onset diabetes or impaired glucose tolerance, and one was divided into two groups based on the different dose of glucocorticoid use. No abnormal blood glucose was found in the other test groups. (Table 3) A total of inclusion was 506, and 246 patients were assigned to the treatment groups, 206 patients were in the control group. The final results showed 19 new-onset diabetes mellitus or impaired glucose tolerance in the trial group and 5 in the control group (3 trials, 95% CI 0.54 to 26.10, p =0.18 I^2^ = 66% Figure 4). It proves patients receiving glucocorticoids therapy had not an increased risk of developing new-onset diabetes mellitus or impaired glucose tolerance. And it seems that there are significant differences in the effect on New-onset diabetes mellitus.

### 3.6. Effect on other adverse effect

We collected data on the effects of glucocorticoids on respiratory infections, and the results are shown four studies reported the number of respiratory infections, and one was divided into two groups based on the different dose of glucocorticoid use. it shows glucocorticoids can increase the risk of respiratory infections (5 trials, 95% CI 0.69 to 3.89, p =0.27 Figure 5). The effect of glucocorticoids on Gastrointestinal SAEs is relatively controversial (4 trials, 95% CI 0.32 to 3.79, p =0.88 I^2^ = 68% Figure 6). Other side reactions were not included in the discussion due to insufficient data or irrelevant with hyperglycemia.

## 4. Discussion

At present, most of the clinical treatment of kidney disease is medium-effect glucocorticoid preparation, namely prednisone, prednisolone and methylprednisolone, which is also reflected in the included studies, and six of the seven groups of data were used with medium-effect glucocorticoid preparation [3]. This is associated with receptor affinity and circadian rhythm of adrenocortical hormone secretion. The physiological, pathological and pharmacological effects of glucocorticoids are mediated by receptors-glucocorticoid receptors. Glucocorticoids easily enter cells through cell membranes and combine with intracellular receptors, thus playing important physiological and pharmacological roles [18]. And because of long-term medication, in order to reduce hormone side effects, it is necessary to choose hormones more in line with circadian rhythm. Another trial selected a novel oral budesonide targeted release agent based on the mechanism by which the mucosal immune system plays a role in IgA nephropathy (IgAN) [19–21].

We found that during the retrieval process, all the nephropathy that met the retrieval criteria were IgAN. IgAN was first reported in 1968 by Dr J. Berger and Hinglais [22]. It is an inflammatory renal disease characterised by the deposition of IgA in the glomerular mesangium [23]. It is known to be the most common form of primary glomerulonephritis throughout the world now [24–27]. Due to the partially unknown pathogenesis, the specific treatment has not been determined. In the last 20 years, a lot of people have tried treatments, and several studies have been published to illustrate their results. According to evidence-based medicine, patients with IgAN with 24 h proteinuria lasting≥1 g and glomerular filtration rate>50 mL/min after 3-6 months of supportive therapy (e. g. target blood pressure achieved with angiotensin converting enzyme inhibitors/angiotensin II receptor antagonists) can receive glucocorticoid therapy for 6 months [28]. As we know, glucocorticoid drug treatment may have certain side effects, such as for blood sugar, because the inhibition of the endogenous pituitary-hypothalamic axis will lead to adrenal atrophy and adrenal cortex dysfunction, produce steroid diabetes, but glucocorticoid for blood sugar and other safety evaluation, is not much. We found that in the published meta analysis, the relationship between glucocorticoid and blood glucose was not explicitly proposed due to the lack of the data included [29].

In this meta-analysis, we identified 7 RCTs that compared the glucocorticoids regimens with control groups. The meta-analysis showed that glucocorticoids were statistically significant in protecting kidney function and reducing proteinuria in patients with renal disease compared with controls. This evidence is fairly clear in the majority of RCTs, even with their quality limitations and heterogeneity, high heterogeneity in proteinuria statistics, possibly with too large number of diseases included in the study, short time, and disturbed by other drugs. According to the 2020 Kidney Disease Improving Global Outcomes (Kidgo) guide, It is recommended that 6-month corticosteroid therapy be considered in IgAN patients who have received optimal treatment but are still at high risk for CKD progression. The data also further illustrate the effectiveness of glucocorticoid therapy. Alternatively, we evaluated the safety of glucocorticoid drugs. Overall, glucocorticoids are well tolerated, with no significant effect on blood glucose. Because some studies (Rauen, T. 2015\Rauen, T. 2018) did not separate new-onset diabetes from abnormal glucose tolerance, subgroup analysis was not possible despite high heterogeneity. However, it can be seen from *p* value that glucocorticoids have no significant relationship with blood glucose. Meanwhile, we find no significant significance for other side reactions such as digestive tract diseases and respiratory tract infections.

Although our analysis has some reference significance for glucocorticoid use, our meta-analysis has several limitations that should be considered. First of all, fewer studies included may lead to a small sample size. In addition, although three of them have a Jaded score of 7 points, the overall quality of the articles is high, but some of the articles are not very good quality, therefore, we conducted a quality assessment of the studies included and clearly showed the details of each study. However, some of the studies do not fully show the details of all the indicators, which may have some impact on our analysis results. Second, the dosage and type of drugs, that is, those used in the glucocorticoid treatment group, varied. At the same time, the primary endpoint of these studies was slightly different, although classified as a decline in renal function, the extent of the decline is still somewhat different. In addition, there are not enough indicators of blood sugar, such as hemoglobin, OGTT, etc., the real results of treatment may be a little deviation. Finally, most studies included patients receiving concomitant drugs, such as RAS blockers, receptor blockers, or calcium channel blockers, which may also be a factor in the high heterogeneity. Although we included this type of study in the intervention and control groups in the same way, further studies are needed to evaluate the effects of glucocorticoid drugs alone on patients who have not received other treatments.

## 5. Conclusion

Compared with control, glucocorticoids seems to be effective and relatively safe for both reducing proteinuria and stabilizing kidney function in patient with renal disease. Glucocorticoids had no significant relationship with blood glucose. Glucocorticoids agents are a promising strategy in curing renal disease. Further clinical studies are warranted to explore the long term efficacy and safety of glucocorticoids.

## Figures and Tables

**Figure 1:** Flow diagram of studies considered for inclusion.

**Figure 2:** Comparison of glucocorticoids versus controls on renal survival.

**Figure 3:** Comparison of glucocorticoids versus controls on daily proteinuria.

**Figure 4:** Comparison of glucocorticoids versus controls on blood glucose.

**Figure 5:** Comparison of glucocorticoids versus controls on respiratory infections.

**Figure 6:** Comparison of glucocorticoids versus controls on Gastrointestinal SAEs.

**Table 1:** Characteristics of interventions and populations at baseline and end of treatment in included RCTs.

RCTs	The primary disease	Drugs		Baseline characteristics	Follow-up months	Treatment group		Control group	
		Treatment group	Control group			Sample sizes	DRF	Sample sizes	DRF
Ronald 2006	IgAN	Prednisone 60 mg/m^2^ every other day for 3 months, and then 40 mg/m^2^ every other day for 9 months, and then 30 mg/m^2^ every other day for 12 months	Placebo	Age<40; renal biopsy showing IgAN; eGFR>50 ml/min per 1. 73m^2^; UPCR≥1. 0 g/g or moderate proteinuria, UP/C ratio ≥0. 5plus renal biopsy changes	24	30	2	29	4
lv 2009	IgAN	Prednisone 0. 8 to 1. 0 mg/kg/d, for 8 weeks, then the dose was tapered by 5 to 10 mg every 2 week	Cilazapril alone	Renal biopsy showing IgAN; age18~65years; urine protein excretion of 1 to 5 g/d; eGFR≥30 mL/min	24	33	1	30	7
Fellström2017	IgAN	TRF-budesonide 16 mg/d and 8 mg/day	Placebo	Persistent proteinuria (UPCR ≥0·5 g/g or proteinuria ≥0·75 g/day); eGFR≥45 mL/min)	9	51(8 mg/d) 49(16 mg/d)	0	50	0
lv 2017	IgAN	Methylprednisolone 0. 6-0. 8 mg/kg/d, then tapered by 8 mg/d each month	Placebo	Proteinuria≥1 g/d and eGFR of 20~120 mL/min	6 ~ 8	136	8	126	20
Rauen, T. 2015	IgAN	Methylprednisolone, administered intravenously at a dose of 1 g per day for 3 days at the start of months 1, 3, and5; oral prednisolone at a dose of 0. 5 mg per kilogram per 48 hours on the other days	Supportive care	Age 18~70 year; proteinuria level above 0. 75 g/d; impaired renal function(eGFR 60-90 mL/min)	6	55	<21	80	22
Rauen, T. 2018	IgAN	Methylprednisolone, administered intravenously at a dose of 1 g per day for 3 days at the start of months 1, 3,and5; oral prednisolone at a dose of 0. 5 mg per kilogram per 48 hours on the other days	Supportive care	GFR>60 ml/min	6	55	12	54	16
Shoji 2000	IgAN	Prednisolone 0. 8 mg/kg/day and tapering to 10 mg q. o. d. 1 year	Dypiridamole 300 mg/day	Proteinuria less than 1. 5 g/day; plasma creatinine concentrations<1. 5 mg/dl. Age 15 and 55 years.	12	11	0	8	0

**Table 2:** Quality assessment of RCTs included in the review.

Included studies	Randomization	Concealment of allocation	Double blinding	Total withdrawals and dropouts	Modified Jadad score (7-point)
Ronald. 2006	2	2	2	1	7
Lv. 2009	2	2	0	1	5
Fellström 2017	2	2	2	1	7
Lv. 2017	2	2	2	1	7
Rauen, T. 2015	2	1	0	1	4
Rauen, T. 2018	2	1	0	1	4
Shoji. 2000	2	0	0	0	2

**Table 3:** Patients of New-onset diabetes mellitus or impaired glucose tolerance.

RCTs	Treatment group		Control group	
	Sample size	New-onset diabetes/impaired glucose tolerance	Sample size	New-onset diabetes/impaired glucose tolerance
Lv 2009	33	0	30	0
Fellström 2017	51(8 mg/d) 49(16 mg/d)	0	50	0
Lv 2017	136	2	126	3
Rauen, T. 2015	55	8	80	1
Rauen, T. 2018	55	9	54	1
Shoji 2000	11	0	7	0

## Data Availability

No data were used to support this study.
